# Ginkgo biloba extract EGb 761–induced upregulation of LincRNA-p21 inhibits colorectal cancer metastasis by associating with EZH2

This article has been retracted.

**DOI:** 10.18632/oncotarget.21345

**Published:** 2017-09-27

**Authors:** Tingting Liu, Junzhong Zhang, Zhongqiu Chai, Gang Wang, Naiqiang Cui, Bing Zhou

**Affiliations:** ^1^ Department of Integrated Chinese and Western Medicine Surgery, Tianjin University of Traditional Chinese Medicine, Tianjin, China; ^2^ Department of Anorectal Surgery, Tianjin Binhai New Area Traditional Chinese Medicine Hospital, Tianjin, China; ^3^ Department of Science and Education, Tianjin Binhai New Area Traditional Chinese Medicine Hospital, Tianjin, China; ^4^ Department of Oncology, Ruijin Hospital of Shanghai Jiaotong University, Shanghai, China

**Keywords:** EGb 761, colorectal cancer, LincRNA-p21, metastasis, EZH2

## Abstract

EGb 761, the standard ginkgo biloba extract, is frequently prescribed in traditional Chinese medicine. Currently, there is no research focusing on its role in human colorectal cancer progression. In our study, we determined the anti-metastatic effect of EGb 761 on colorectal cancer cells and further explored the potential underlying regulatory mechanism. The cell migration and invasion assay indicated that EGb 761 treatment of colorectal cancer cells induced inhibition of cell migration and invasion ability in a concentration-dependent manner. To further explore the underlying regulatory mechanisms that may account for these findings, we performed quantitative real-time PCR (RT-qPCR), western blotting and immunoprecipitation analysis. The results showed that EGb 761 induced upregulation of LincRNA-p21 expression in a dose- and time-dependent manner. Overexpression of LincRNA-p21 also suppressed colorectal cancer cell metastasis. Furthermore, EGb 761 as well as LincRNA-p21 inhibited the expression of extracellular matrix protein, fibronectin. More importantly, RNA immunoprecipitation (RIP) and Chromatin immunoprecipitation (ChIP) assays showed that LincRNA-p21 directly interacted with EZH2, and this interaction suppressed the expression of fibronectin. Finally, the gain and loss function assay revealed that EGb 761 inhibited migration, invasion and fibronctin expression by the LincRNA-p21/EZH2 pathway in colorectal cancer cells. Hence, EGb 761 may be a promising treatment regimen for colorectal cancer and restoration of LincRNA-p21 levels may be helpful for enhancing the anti-cancer effect of EGb 761.

## INTRODUCTION

Colorectal cancer is associated with high mortality, and is one of the most general malignant cancers in digestive system [1]. Cell migration and invasion are fundamental properties of progressive colorectal cancer, and metastasis is the major cause of death for patients with CRC and increases the risk of tumor recurrence [2]. Currently, surgery resection with subsequent chemotherapy is still the most commonly used method for colorectal cancer. However, a large proportion of patients receiving chemotherapy finally become metastatic and chemoresistant, and this has been a key barrier to the efficacy of colorectal cancer treatment [3]. Thus, revealing the underlying mechanism and finding new therapeutic approaches are necessary for developing effective therapies for colorectal cancer patients.

Plants have provided a rich source of therapeutic agents and bases for synthetic drugs. It is believed that herbage may have pharmaceutical composition, which can be used for clinical practice, such as ginkgo biloba [4]. The extracts of ginkgo biloba are widely used for the supplements of sold herbal. The standard ginkgo biloba extract EGb 761, which contains 24% ginkgo lavone glycoside and 6% terpene lactones, is one the most important antioxidant properties [5]. Several studies have reported that the antioxidant activity of Ginkgo biloba extract could be helpful in the prevention and therapy of diseases and degenerative processes associated with oxidative stress [6–8]. In addition, EGb 761 was also reported to have anti-tumor function in various cancers, including ovarian cancer, hepatocellular cancer and oral cavity cancer [9–11]. However, the anti-tumor effect of EGb 761 on colorectal cancer is still not well known.

During the past decade, large-scale sequencing efforts and the ENCODE project have revealed that a large fraction of the human noncoding genome is transcribed [12]. Long non-coding RNAs (lncRNAs) are defined as transcripts > 200 nucleotides in length and have been implicated in a variety of physiological and pathological processes [13]. In cancer, aberrant expression and mutations of lncRNAs can contribute to tumor development and progression by promoting proliferation, invasion, metastasis, and survival [14, 15]. Long intergenic non-coding RNA-p21 (LincRNA-p21) (3100 nt) is located on chromosome 6, approximately 15 kb upstream from the Cdkn1a (p21) gene [16]. LincRNA-p21 was first reported to be a direct transcriptional target of p53 and to mediate p53-dependent apoptosis in doxorubicintreated mouse embryo fibroblasts (MEFs) (16). Another more recent report indicates that LincRNA-p21 derails somatic cell reprogramming by sustaining H3K9me3 and CpG methylation at pluripotency gene promoters [17].

In this report, we investigated the effect of EGb 761 on colorectal cancer metastasis and the underlying regulatory mechanism. We found that EGb 761 suppressed colorectal cancer cell metastasis in a dose-dependent manner. More importantly, EGb 761 treatment promoted the expression of LincRNA-p21, and this upregulation of LincRNA-p21 eventually suppressed colorectal cancer cell migratory and invasive capacity through associating with EZH2.

## RESULTS

### EGb 761 inhibits the migration and invasion of colorectal cancer cells

We firstly evaluated the effect of EGb 761 on colorectal cancer cell metastasis. Wound-healing assay and Matrigel invasion assay were used to detect the migratory and invasive capacity of colorectal cancer cells, respectively. As shown in Figure 1A, EGb 761 treatment significantly inhibited the migration of SW480 and SW620 cells in a dose-dependent manner. Additionally, the invasive capacity was also dramatically inhibited after treatment of EGb 761 at the concentration of 250 and 500 mg/L in both noninvasive cell line SW480 and invasive cell line SW620 (Figure 1B). Moreover, the number of cells went through the membrane in the 500 mg/L group was significantly lower than that in group of cells treated with 250 mg/L of EGb 761 in both cell lines. Interestingly, CCK8 assay indicated that EGb 761 treatment had no significant effect of cell viability in both SW480 and SW620 cells (date not shown), which excludes the interference of EGb 761-induced cell cytotoxic effect.

**Figure 1:** EGb 761 inhibits the migration and invasion of colorectal cancer cells **(A)** Wound-healing assay indicated that EGb 761 treatment inhibited the migratory capacity of SW480 and SW620 cells in a dose-dependent manner. **(B)** Matrigel invasion assay revealed that EGb 761 suppressed the invasive capacity of SW480 and SW620 cells in a dose-dependent manner.

### Identification of candidate lncRNAs by high-throughput Hiseq sequencing

After having revealed the anti-metastatic effect of EGb-67, we further explored the underlying mechanism that may explain the observations. Various reports have indicated that lncRNA may participate in cancer progression and chemoresistance [18–20]. To identify the potential lncRNAs that may act as critical regulators during the function of EGb 761, e performed high-throughput HiSeq sequencing by extracting the total RNA from SW480 cells treated with 500 mg/L EGb 761 and SW480 cells free of treatment of EGb 761. The expression of 75 lncRNAs showed more than 2-fold difference between EGb 761 treated SW480 cells and control cells (Figure 2). Among these, 34 lncRNAs was up-regualted in EGb761 treated cells when compared with control cells. The lncRNA MAGI2-AS3 showed the highest expression with 128.6347 fold higher, followed by LincRNA -p21 and LOC645166. There were 41 lncRNAs that showing significant down-regulated expression level. Of these, lncRNA ZNF37BP showed the most decreased expression (95.9948 times lower), followed by LOC389906 and TDRG1 (Table 1).

**Figure 2:** The heat map shows expression of the 75 lncRNAs that showed more than 2-fold difference between EGb 761 treated SW480 cells (8 samples) and control cells (8 samples) The heat map was generated with an R package using normalization across rows (cells). T: SW480 EGb 761 treated cells; C: SW480 control cells.

**Table 1:** Candidate lncRNAs selected on a basis of the Hiseq analysis

Seqname	Location	Regulation (T vs C)	Fold change	*P* value
MAGI2-AS3	Chr7q21.11	Up	78.6347	0.00017490
LincRNA-p21	Chr6p21.2	Up	55.3165	0.00027656
LOC645166	Chr1q21.1	Up	39.1768	0.00052836
ZNF37BP	Chr10q11.21	Down	95.9948	0.00008362
LOC389906	ChrXp22.33	Down	54.8693	0.00030942
LINC00189	Chr6p21.2	Down	41.6396	0.00048731

T: EGb 761 treated cells; C: control cells.

### LincRNA-p21 was induced by EGb 761 treatment in colorectal cancer cells

We then performed RT-qPCR to verify the potential differentially expressed lncRNAs, and the results showed that LincRNA-p21 expression was significantly increased in EGb 761 treated SW480 cells when compared with control cells, while the other five lncRNAs showed no statistical significance (Figure 3A-3F). Recent studies indicated that LincRNA-p21 is an lncRNA associated with colorectal cancer and metastasis [21, 22]. Therefore, we think that EGb 761 may upregulate LincRNA-p21 to suppress colorectal cancer metastasis. The RT-qPCR assay showed that LincRNA-p21 was downregulated in primary colorectal cancer tissues when compared with noncancerous tissues (Figure 3G). Similarly, LincRNA-p21 was also downregulated in SW480 and SW620 cells when compared with normal colon cell line FHC (Figure 3H). More importantly, the expression of LincRNA-p21 was significantly increased in colorectal cancer cells treated with EGb-761 in both dose-dependent and time-dependent manner (Figure 3I).

**Figure 3:** LincRNA-p21 was induced by EGb 761 treatment in colorectal cancer cells **(A-F)** Concentrations of the six identified lncRNAs in SW480 EGb 761 treated cells and control cells using RT-qPCR assay. **(G)** RT-qPCR showed that the expression of LincRNA-p21 was significantly downregulated in primary colorectal cancer tissues when compared with noncancerous tissues. **(H)** LincRNA-p21 was also downregulated in SW480 and SW 620 cells when compared with normal normal colonic cell line FHC. **(I)** EGb 761 induced the expression level of LincRNA-p21 in a dose- and time-dependent manner. Error bars represent median ± SD. ^**^P<0.01.

### EGb 761 inhibits metastasis of colorectal cancer cells through upregulation of LincRNA-p21

The effect of LincRNA-p21 on cell metastasis was then evaluated. As expected, overexpression of LincRNA-p21 with p-LincRNA-p21 significantly suppressed migratory and invasive capacity of SW480 and SW620 cells (Figure 4A and 4B). Then, LincRNA-p21 was silenced by si-LincRNA-p21. Figure 3C indicated that the si-LincRNA-21 #3 showed a best knockdown effect compared with the si-LincRNA-p21 #1 and si-LincRNA-p21 #2, and si-LincRNA-p21 #3 was chosen for further experiments. The gain and loss function assay showed that knockdown of LincRNA-p21 dramatically reversed the effect of EGb 761 on colorectal cancer cell invasion (Figure 4D).

**Figure 4:** EGb 761 inhibits metastasis of colorectal cancer cells through upregulation of LincRNA-p21 **(A-B)** Overexpression of LincRNA-p21 suppressed migration (A) and invasion (B) of SW480 and SW620 cells. **(C)** LincRNA-p21 was silenced by specific siRNAs. **(D)** EGb 761 treatment significantly inhibited the invasive capacity of colorectal cancer cells, however, this effect was dramatically reversed by co-transfection of si-LincRNA-p21. **(E)** Western blot experiments indicated that EGb 761 as well as LincRNA-p21 treatment significantly inhibited the expression of fibronectin in colorectal cancer cells. Error bars represent median ± SD. ^*^P<0.05, ^**^P<0.01.

One of the most important causes of enhanced cell metastasis is the accumulation of extracellular matrix regulators such as fibronectin. Thus we detect the effect of EGb 761 and LincRNA-p21 on fibronectin expression. Western blot experiments indicated that EGb 761 as well as LincRNA-p21 treatment significantly inhibited the expression of fibronectin in colorectal cancer cells (Figure 4E), indicating that EGb 761 may regulate colorectal cancer cell metastasis through inhibiting fibronectin expression.

### LincRNA-p21 interacts with EZH2 in colorectal cancer cells

Previous studies indicated that LincRNA-p21 functioned as an tumor suppressor gene through participation in epigenetic regulation, such as histone methylation and/or CpG methylation at pluripotency gene promoters [17]. It is known that EZH2, working with EED and SUZ12, the other two essential components of the Polycomb repressive complex2 (PRC2), functions primarily as a methyltransferase catalyzing histone H3 lysine 27 trimethylation (H3K27me3) and promoting gene silencing. To validate the interaction between LincRNA-p21 and EZH2, we performed RNA immunoprecipitation (RIP) assay by using EZH2 antibody to concentrate LincRNA-p21 in colorectal cancer cells. As expected, a significant enrichment of LincRNA-p21 with EZH2 antibody was observed when compared with the non-specific IgG antibody. These results were confirmed by using another primer pair for LincRNA-p21 (Figure 5A), but no enrichment of β-actin or lncRNA control was confirmed in SW480 cells (Figure 5B). Subsequently, RNA pulldown was done to determine the the direct interaction between the two molecules. Compared with lncRNA control, a significant increased enrichment of EZH2 was identified by LincRNA-p21 (Figure 5C). Collectively, we validated that LincRNA-p21 can directly interact with EZH2 in colorectal cancer.

**Figure 5:** LincRNA-p21 is associated with EZH2 in colorectal cancer **(A)** RIP experiments were performed using the EZH2 antibody to immunoprecipitate RNA and two primers to detect LincRNA-p21, and a relatively high enrichment of LincRNA-p21 was found compared with IgG control. **(B)** RIP experiments showed that no enrichment of β-actin or lncRNA control was confirmed in SW480 cells. **(C)** Biotinylated LincRNA-p21 or control were incubated with nuclear extracts (SW480 and SW620 cells), targeted with streptavidin beads and associated proteins were resolved in a gel. Western blotting analysis of the specific association of EZH2 and LincRNA-p21 was performed. Error bars represent median ± SD. ^*^P<0.05.

### LincRNA-p21 represses fibronectin expression by associating with EZH2

Based on the above observations, we sought to determine whether the negative regulation of fibronectin expression by LincRNA-p21 is through association with EZH2. EZH2 was silenced by transfection with si-EZH2 (Figure 6A), and the silence of EZH2 significantly increased fibronectin expression levels in SW480 and SW620 cells (Figure 6B and 6C). To further address how LincRNA-p21 is involved in fibronectin regulation through the enrichment of EZH2, we used ChIP analysis to determine the effect of p-LincRNA-p21 on histone modification in the fibronectin promoter with an anti-H3K27-me3 antibody in SW480 cells. Specific primers were designed to detect the sequences that immunoprecipitated by H3k27me3 or EZH2 on the promoter region of fibronectin gene (Figure 6D). The enrichment levels of EZH2 and H3K27-me3 were significantly increased in LincRNA-p21-overexpressed cells compared to control cells (Figure 6E and 6F), while enrichment of IgG with firbonectin promoter showed no significant change after overexpression of LincRNA-p21 (Figure 6G). This suggests that LincRNA-p21 inhibits fibronectin expression through associating with EZH2 and specific binding to fribronctin gene promoter region.

**Figure 6:** LincRNA-p21 represses fibronectin expression by associating with EZH2 **(A)** Specific siRNA targeting EZH2 (si-EZH2) significantly silenced EZH2 mRNA expression in colorectal cancer cells. **(B-C)** Knockdown of EZH2 significantly promoted fibronectin expression in both transcript (B) and protein level (C). **(D-G)** ChIP analysis of SW480 cells treated with p-LincRNA-p21 was conducted on fibronectin promoter (primer a-c) and GAPDH promoter (primer d-e) regions using the indicated antibodies. Enrichment was determined relative to input controls. These results show data from at least three independent experiments. Error bars represent median ± SD. ^*^P<0.05, ^**^P<0.01.

### EGb 761 suppresses the metastatic capacity of colorectal cancer cells by LincRNA-p21/EZH2 pathway

The biologic consequences of LincRNA-p21 and EZH2 in EGb 761 regulation of migration and invasion were then examined using gain and loss functional assays. As shown in Figure 7A, EGb 761-induced inhibition of fibronectin transcript expression was potently relieved by LincRNA-p21 or EZH2 silencing in SW480 cells. Consistent with the above results, LincRNA-p21 or EZH2 silencing also reversed fibronectin protein level in SW480 cells treated with EGb 761 (Figure 7B). Scratch assays showed that EGb 761-induced suppression of cell migration is partially abolished by LincRNA-p21 or EZH2 knockdown in SW480 and SW620 cells (Figure 7C). Additionally, Matrigel invasion assay showed that LincRNA-p21 or EZH2 knockdown significantly rescued EGb 761-induced inhibition of cell invasion in both SW480 and SW620 cell lines (Figure 7D). To conclude, we finally demonstrated that EGb 761 induces the metastatic ability of colorectal cancer cells through a LincRNA-p21/EZH2 signaling pathway.

**Figure 7:** EGb 761 inhibits migration and invasion of colorectal cancer cells by LincRNA-p21/EZH2 pathway **(A-B)** EGb 761-induced inhibition of fibronectin mRNA (A) and protein (B) expression was potently relieved by LincRNA-p21 or EZH2 silencing in SW480 cells. **(C)** Wound-healing assay indicated that EGb 761-induced suppression of cell migration is partially abolished by LincRNA-p21 or EZH2 knockdown in SW480 and SW620 cells. **(D)** Matrigel invasion assay showed that LincRNA-p21 or EZH2 knockdown significantly rescued the EGb 761-induced inhibition of invasive capacity compared with control in both SW480 and SW620 cells. Error bars represent median ± SD. ^*^P<0.05.

## DISCUSSION

Although there have been inroads into the treatment of colorectal cancer [23, 24], these treatment strategies often cause resistance and bring side effects with marginal results. Many patients therefore turn to alternative treatment [25]. EGb 761 is thought to have important biological functions and medicinal effects in various processes, such as inflammatory reaction, angiogenesis and initiation and progression of tumors [10]. In the present study, we investigated the effect of EGb 761 on colorectal cancer cell metastasis and further explored the underlying regulatory mechanism. We found that EGb 761 suppressed migration and invasion of colorectal cancer cells through the inhibition of fribronectin expression by LincRNA-p21/EZH2 pathway.

Those patients succumb to their disease mostly for the reason of chemoresistance, and invasion and spread of solid tumors are the major causes of chemoresistance in patients with CRC [26]. The Chinese traditional medicine EGb 761 has not been applied in the clinical practice, yet its anti-cancer effect has been well investigated on cancer proliferation, apoptosis and cell cycle regulation [27, 28]. However, its role in colorectal cancer metastasis is not well known. Our preliminary date revealed that EGb 761 can significantly inhibited the migratory and invasive capacity of colorectal cancer cells. It is well known that searching new therapeutic approach and targets, and better understanding the pathway related to EMT is essential for improving the prognosis of CRC patients. LincRNA-p21 is a lncRNA that associates with regulation of cancer metastasis and colorectal cancer progression. Jia et al demonstrated that lincRNA-p21 inhibits invasion and metastasis of hepatocellular carcinoma through Notch signaling-induced epithelial-mesenchymal transition [22]. Wang et al found that LincRNA-p21 suppressed metastasis and promoted the clinical survival rate of patients with colorectal cancer through improving the therapeutic efficacy and suppressing the proteins involved in Wnt/β-catenin regulatory pathway [21]. These suggest that LincRNA-p21 may be a critical regulatory factor during the EGb 761-induced anti-metastatic process. As expected, we found that LincRNA-p21 was induced by EGb 761 treatment and knockdown of LincRNA-p21 dramatically reversed the effect of EGb 761 on cell metastasis in colorectal cancer. More importantly, we revealed that EGb 761 as well as LincRNA-p21 inhibited the expression of fibronectin, a important extracellular matrix protein, which may explain the functional role of EGb 761 and LincRNA-p21 in colorectal cancer metastasis.

We attempted to unravel the molecular switch of EGb 761 and LincRNA-p21 controlling this malignant phenotype and elucidate the underlying mechanisms on the metastatic evolution of colorectal cancer. EZH2 is a pivotal enzyme in histone modification that plays a key role in catalyzing H3K27me3, resulting in transcriptional silencing of target genes [18]. For example, studies have suggested that EZH2 can inhibit E-cadherin expression through this methylation, thereby increasing cancer invasiveness and metastasis [29–31]. On the other hand, Akizu et al found that EZH2 can regulate neuroepithelium structure and neuroblast proliferation by repressing p21 [32], suggesting the interaction between LincRNA-p21 and EZH2 may be important. By performing RIP experiment and RNA pulldown assay, we found that LincRNA-p21 can directly interact with EZH2, suggesting a novel potential role of LincRNA-p21/EZH2 pathway during EGb 761 functioning.

It is widely accepted that EZH2 is an important epigenetic regulatory factor by mediating modifications in histone methylation resulting in the repression of numerous tumor suppressor or promoter genes [18]. One of the most important causes of enhanced cell metastasis is the formation of EMT process and the subsequent accumulation of extracellular matrix regulators, such as fibronectin [33, 34]. To determine whether LincRNA-p21/EZH2 influence the expression of fibronectin, we performed ChIP assay and found that LincRNA-p21 decreased fibronectin expression through EZH2 mediating H3K27me3 formation in colorectal cancer. As fibronectin can enhance cell migration, this inhibition of fibronectin by LincRNA-p21/EZH2 can lead to the suppression of cancer cell metastasis. Additionally, silence of EZH2 significantly increased fibronectin expression levels in SW480 and SW620 cells, which further confirmed the direct interaction between EZH2 and fribronectin. Collectively, we revealed that LincRNA-p21 can inhibit fibronectin expression through associating with EZH2 and specifically binding to fribronctin gene promoter region.

Take a step further, we eventually sought to identify whether EGb 761 regulates colorectal cancer metastasis and fibronectin expression by a LincRNA-p21/EZH2 pathway. Co-transfection assay showed that knockdown of LincRNA-p21 or EZH2 partially reversed the inhibitory effect of EGb 761 on firbonectin expression in both transcript and protein level. Similarly, scratch assay and Matrigel invasion assay showed that LincRNA-p21 or EZH2 knockdown dramatically abrogated the EGb 761-induced promotion of cell migration and invasion capacity in both colorectal cell lines.

In conclusion, our integrated approach demonstrated that EGb 761 can suppress fibronctin expression and metastatic capacity in colorectal cancer. The mechanistic research indicated that EGb 761 inhibited migration, invasion and fibronctin expression by LincRNA-p21/EZH2 pathway in colorectal cancer. Hence, EGb 761 could serve as a promising treatment regimen for patients with colorectal cancer, and restoration of LincRNA-p21 levels may be helpful for enhancing the anti-cancer effect of EGb 761.

## MATERIALS AND METHODS

### Patient samples

Sixty-six cancer tissues and paired adjacent noncancerous tissues (male/female: 44/22, range of age: 47-78) from primary colorectal cancer patients were collected at Tianjin Binhai New Area Traditional Chinese Medicine Hospital between 2014 and 2016. All the patients were pathologically confirmed and the tissues were collected immediately after they were obtained during the surgical operation, and then stored at -80°C to prevent RNA loss. They were classified according to the World Health Organization (WHO) criteria and staged according to the tumor-node-metastasis (TNM) classification. Written informed consent was obtained from all patients according to the guidelines approved by the Ethics Committee of Tianjin Binhai New Area Traditional Chinese Medicine Hospital.

### HiSeq sequencing

Total tissue RNA was extracted by one-step extraction using a Trizol kit (Life Technologies, USA), and the purity and quantity of RNA were determined by UV spectrophotometry. cDNA library construction and sequencing were performed according to previously described methods [35]. Briefly, after extraction of total RNA, ribosomal RNA was separated to isolate as ncRNA as possible. RNA containing poly(A) was then removed. RNA fragments were broken into short fragments randomly. The first chain of cDNA was generated using RNA fragments as templates and 6-bp random primers. Second chain of the cDNA was synthesized according to the kit’s instruction (TakaRa Co., Ltd., Dalian, China). After purification, end repair, base A and sequencing joint adding, the generated cDNA was fragmented using uracil-N-glycosylase (UNG). cDNA fragments were chosen according to size, then PCR amplification was performed to establish the complete sequencing cDNA library. lncRNAs were sequenced using the high-throughput, high-sensitivity HiSeq 2500 sequencing platform (Illumina Company, USA). The whole process and subsequent data analysis were performed by Kangchen Bio-tech, Shanghai P.R. China. FastQC software was used for quality control of the pretreated data.

### Cell culture

The human colorectal cancer cell lines SW480, SW620 and human fetal normal colonic cell (FHC) were obtained from the Type Culture Collection of the Chinese Academy of Sciences (Shanghai, China) in 2014. All colorectal cancer cell lines were maintained in RPMI 1640 (Thermo Fisher Scientific, Wilmington, DE, USA) containing 10% fetal bovine serum (FBS) (Sigma-Aldrich, St. Louis, MO, USA), 100 U/ml penicillin, and 100 g/ml streptomycin (Life Technologies, Grand Island, NY, USA) at 37°C in 5% CO_2_ and 95% air. Normal colon FHC cells were grown in Dulbecco’s Modified Eagle’s Medium (DMEM)/F12 medium with 10% FBS, 10 ng/mL cholera toxin, 5 μg/mL transferrin, 5 μg/mL insulin, 100 ng/mL hydrocortisone and an extra 10 mM of 4-(2-hydroxyethyl)-1-piperazineëthanesulfonic acid (HEPES) at 37°C in 5% CO_2_ and 95% air. The cells were incubated with various concentrations (0-500 mg/L) of standard Ginkgo biloba extract solution (EGb 761, Dr. Willmar Schwabe Pharmaceuticals, Karlsruhe, Germany) for 24 or 48 h. The cell authenticity was determined by short tandem repeat analysis technology (Cell ID™ System, Promega, Madison, WI).

### Cell transfection

The small interfering RNAs (siRNA) that specifically target human LincRNA-p21 and EZH2 were designated as si-LincRNA-p21 and si-EZH2 (Genechem corporation, Shanghai, China). The LincRNA-p21 overexpression plasmid (p-LincRNA-p21) or control vector (p-Vector) was purchased from Addgene. Colorectal cancer cells were plated in 24-well plates at 1 × 10^5^ per well. Forty-eight hours after plating, 100 nM of RNA oligoribonucleotides were transfected into the cells with Lipofectamine 2000 (Invitrogen, Carlsbad, CA, USA) according to the manufacturer’s instructions.

### Total RNA and protein extraction

Total RNA was isolated from primary tumor tissues or colorectal cancer cell lines using TRIzol reagent (Invitrogen). The extracted total RNA was eluted in 20 μl nuclease-free water, and the RNA concentration was measured by Nanodrop 2000 (Thermo Fisher Scientific). For protein extraction, cells were lysed with radioimmunoprecipitation assay (RIPA) buffer (Sigma-Aldrich) containing protease inhibitors (Sigma-Aldrich). Protein quantification was done using a BCA protein assay kit (Thermo Fisher Scientific).

### Reverse transcription and quantitative real-time PCR (RT-qPCR)

The cDNA was synthesized from 200 ng extracted total RNA using the PrimeScript RT reagent Kit (Takara Bio Company, Shiga, Japan) and amplified by RT-qPCR with an SYBR Green Kit (Takara Bio Company) on an ABI PRISM 7500 Sequence Detection System (Applied Biosystems) with the housekeeping gene GAPDH as an internal control. The 2^-ΔΔCt^ method was used to determine the relative quantification of gene expression levels. All the premier sequences were synthesized by RiboBio (Guangzhou, China), and their sequences are shown in Table 2.

**Table 2:** Information of the RT-qPCR primer sequence and siRNA sequence

RT-qPCR primer name	Primer sequences (5’-3’)
LincRNA-p21 (Forward)	CCCGGGCTTGTCTTTTGTT
LincRNA-p21 (Reverse)	GAGTGGGTGGCTCACTCTTCTG
EZH2 (Forward)	GGCTCCTCTAACCATGTTTACAACT
EZH2 (Reverse)	AGCGGTTTTGACACTCTG AACTAC
Fibronectin (Forward)	TCT TCCAGGAACCTCTGTGATG
Fibronectin (Reverse)	CAATGCCGCCATCGCTTACACC
GAPDH (Forward)	GCACCGTCAAGGCTGAGAAC
GAPDH (Reverse)	ATGGTGGTGAAGACGCCAGT
**ChIP-qPCR primer name**	**Primer sequences (5’-3’)**
Fibronectin-a (Forward)	TGGATCATCTGAGGACAGGA
Fibronectin-a (Reverse)	CCACCACGACTGGCTAATTT
Fibronectin-b (Forward)	AGTCCCACAACAGCATAGGG
Fibronectin-b (Reverse)	TCCCTAGGTCAGGACCACCT
Fibronectin-c (Forward)	CTCCAGCTTGGGTGAAAGAG
Fibronectin-c (Reverse)	GGGCTTTTACACTTGGCTAG
GAPDH-d (Forward)	AGGGAAGCTGACAGGGATGGCG
GAPDH-d (Reverse)	ATCGAAGATGGACGAGTGGGTA
GAPDH-e (Forward)	CCCCGCTACTCCTCCTCCTAAG
GAPDH-e (Reverse)	TCCACGACCAGTTGTCCATTCC
**siRNA name**	**siRNA sequences (5’-3’)**
si-LincRNA-p21 #1	UGAAAAGAGCCGUGAGCUAdTdT
si-LincRNA-p21 #2	AAATAAAGATGGTGGAATGdTdT
si-LincRNA-p21 #3	CUGCAAGGCCGCAUGAUGAdTdT
si-EZH2	AUCAGCUCGUCUGAACCUCUUdTdT
si-NC (GFP)	GGCUACGUCCAGGAGCGCACCdTdT

### Wound-healing assays

Transfected/treated cells were seeded in 6-well plates and cultured to near confluence. Artifcial wounds were created on the cell monolayer using cultureinserts for live cells analysis, and then migrated cells and wound healing were visualized. For each group, at least 3 artifcial wounds were photographed immediately and at the time points indicated after the wound formation. After the wounds were created, the cells were incubated in culture medium without FBS and then photographed at 48 h. Percent of wound closure was calculated with Image J 1.47 software. Each experiment was performed in triplicate.

### Matrigel invasion assays

Cell invasive ability was detected by using Transwell permeable supports (Corning, USA) according to manufacturer’s protocol. Briefly, the transfected/treated cells were plated onto a Matrigel-coated membrane in the upper chamber of a 24-well insert containing medium free of serum. The bottom chamber contained RPMI 1640 with 10% FBS. Cells were incubated at 37°C with 5% CO_2_ for 48 h after plating. Then, the bottom of the chamber insert was fixed with methanol and stained with DAPI. The number of cells that invaded through the membrane was determined from digital images captured on an inverted microscope and calculated with Image J 1.47 software. Each experiment was performed in triplicate.

### RNA immunoprecipitation (RIP)

RIP experiment was performed to investigate whether ribonucleoprotein (RNP) complex contained LincRNA-p21 and its potential binding protein (EZH2) in colorectal cancer cells. The Magna RIP RNA-Binding Protein Immunoprecipitation Kit (Millipore, Bedford, MA, USA) was used according to the manufacturer’s instructions. The RNAs were immunoprecipitated using anti-EZH2 (catalog#4905S, Cell Signaling Technology, Beverly, MA, USA) antibody. Total RNA and controls were also assayed to demonstrate that the detected signals were from RNAs specifically binding to EZH2. The final analysis was performed using RT-qPCR and shown as the fold enrichment of LincRNA-p21. The RIP RNA fraction Ct value was normalized to the input RNA fraction Ct value. Primers are listed in Table 1.

### Chromatin immunoprecipitation (ChIP)

ChIP was performed using the EZ ChIP™ Chromatin Immunoprecipitation Kit (Millipore) according to the manufacturer’s protocol. Briefly, cross-linked chromatin was sonicated into 200-1000 bp fragments. The chromatin was immunoprecipitated using anti-EZH2 (#4905S, Cell Signaling Technology) and anti-H3K27me3 (#07-449, Millipore) antibodies. Normal human immunoglobulin G (IgG) was used as a negative control. RT-qPCR was conducted to detect the relative enrichment according to the method described above. Primers are listed in Table 1.

### Western blot and antibodies

A total of 25 μg protein from each sample was separated on 10% Bis-Tris polyacrylamide gel through electrophoresis and then blotted onto polyvinylidene fluoride (PVDF) membranes (GE Healthcare, Piscataway, NJ, USA). Then, the membrane was blocked with 5% (5 g/100 mL) nonfat dry milk (Bio-Rad, CA, USA) in tri-buffered saline plus Tween (TBS-T) buffer for 2 h. Blots were immunostained with primary antibody at 4°C overnight and with secondary antibody at room temperature for 1 h. Immunoblots were visualized using Immobilon™ Western Chemiluminescent HRP Substrate (Millipore). The primary antibodies used for western blotting were rabbit rabbit anti-human Fibronectin antibody (#sc-8422, 1:1000, Santa Cruz Biotechnology, Santa Cruz, CA, USA), and rabbit anti-human β-actin antibody (#sc-47778, 1:1000; Santa Cruz Biotechnology). Horseradish peroxidase-conjugated (HRP) anti-rabbit antibodies (1:5000; Santa Cruz Biotechnology) were used as the secondary antibodies. Protein levels were normalized to β-actin.

### Statistical analysis

Kolmogorov-Smirnov test was used to determine the normality of the distribution of data in each group. Data were presented as median (interquartile range). Mann-Whitney U test or Kruskal-Wallis test was employed to compare differences of LincRNA-p21 among different groups. Analyses were performed with SPSS version 19.0 software (SPSS, Chicago, IL, USA). Error bars in figures represent SD (Standard Deviation), and statistical significance was defined as two-sided P value < 0.05.
